The article "Nonlinear Dynamic Analysis of Bistable Piezoelectric Energy Harvester with a New-Type Dynamic Amplifier" was published in 2022. Journal: Comput Intell Neurosci.

# Nonlinear Dynamic Analysis of Bistable Piezoelectric Energy Harvester with a New-Type Dynamic Amplifier

**DOI:** 10.1155/2022/7155628

**Published:** 2022-06-25

**Authors:** Dawei Man, Gaozheng Xu, Huaiming Xu, Deheng Xu, Liping Tang

**Affiliations:** ^1^School of Civil Engineering, Anhui Jianzhu University, Hefei 230601, China; ^2^BIM Engineering Center of Anhui Province, Hefei 230601, China

## Abstract

A distributed parametric mathematical model of a new-type dynamic magnifier for a bistable cantilever piezoelectric energy harvester is proposed by using the generalized Hamilton principle. The new-type dynamic magnifier consists of a two-spring-mass system, one is placed between the fixed end of the piezoelectric beam and the L-shaped frame, and the other is placed between the L-shaped frame and the base structure. We used the harmonic balance method to obtain the analytical expressions for the steady-state displacement, steady-state output voltage, and power amplitude of the system. The effect of the distance between the magnets, the spring stiffness ratio and mass ratio of the two dynamic magnifiers, and the load resistance on the performance of the harvester is investigated. Analytical results show that compared with the bistable piezoelectric energy harvester with a typical spring-mass dynamic magnifier, the proposed new-type energy harvester system with a two-spring-mass dynamic magnifier can provide higher output power over a broader frequency band, and increasing the mass ratio of the magnifier tip mass to the tip magnet can significantly increase the output power of the BPEH + TDM system. Properly choosing the stiffness ratio of the two dynamic amplifiers can obviously improve the harvested power of the piezoelectric energy harvester at a low excitation level.

## 1. Introduction

In recent years, the rapid development of wireless sensor networks in building structure health and environmental monitoring has put forward higher requirements for the sustainability of its power supply. Piezoelectric energy harvesting technology is one of the most commonly used energy harvesting technologies, which collects vibration energy from the surrounding environment and converts it into useable energy [1, 2]. In the early stages, different types of linear resonant piezoelectric energy harvesters were designed to generate electrical energy from ambient vibrations. The electro-mechanical coupling equation of a linear cantilever piezoelectric energy harvester was derived and experimentally validated by Erturk and Inman [3, 4]. The ambient vibration excitation frequency usually has the characteristics of time-varying and broadband, so if the ambient vibration frequency does not match the harvester's resonant frequency, the efficiency of the linear piezoelectric energy harvester is not high [5–9]. This makes it difficult to meet the requirements of the practical application for this linear piezoelectric energy harvester [10].

The nonlinear techniques enable piezoelectric energy harvesters to achieve energy harvesting in a wider frequency band. Due to the increase of the working frequency bandwidth, the nonlinear piezoelectric energy harvester is less sensitive to the change of the external excitation frequency than the linear piezoelectric energy harvester and is more suitable for harvesting energy from the ambient vibration in practical applications [11–14]. The nonlinearity of piezoelectric energy harvesters induced by magnetic forces is usually classified into three main categories, namely, monostable [15, 16], bistable [17, 18], and tristable [19, 20]. Bistable piezoelectric energy harvesters (2 stable and 1 unstable equilibrium positions) have been extensively investigated and their broadband advantages over linear energy harvesters have been verified in simulations and experiments [21, 22]. Stanton et al. [23] established an analytical model of a bistable piezoelectric energy harvester consisting of a permanent magnet and a piezoelectric cantilever beam and investigated the dynamic characteristics of the system using numerical simulations and experimental methods. Stanton et al. [24] studied the voltage output of a bistable cantilever piezoelectric energy harvester system under different excitation intensity and analyzed the influence of magnet spacing on the system response. He and Daqaq [25] investigated the influence mechanism of asymmetric potential well characteristics on bistable piezoelectric energy harvester under white noise excitation. Kim et al. [26] proposed an electro-mechanical coupling equation for a hysteresis reversible magneto-elastic piezoelectric energy harvester, and the analytical solutions of the system response are obtained by the multiscale method and the high-dimensional harmonic balance method, respectively. The operating bandwidth and output power of the bistable piezoelectric energy harvester have been substantially increased after entering the interwell motion. However, it requires higher excitation strength. If the excitation strength is low, the bistable energy harvester may exhibit intrawell motion which greatly reduces the output performance of the system [27].

To improve the output performance of the bistable energy harvester under low-level excitation, researchers try to make it easier to oscillate with large amplitude interwell motion. Sebald et al. [28, 29] found that external intervention and increasing the excitation amplitude can help the bistable energy harvester jump from intrawell motion to large amplitude interwell motion. However, the excitation level of the vibration in the real environment is low, and it is difficult to enter the large-scale interwell movement [30]. Ma et al. [31] proposed an asymmetric tristable energy harvester, which has a shallower and wider potential well, so that it can extract vibration energy in a wider frequency range, even at a relatively low excitation level, but the interwell output power amplitude is low in this case. Wang et al. [32] propose a configuration that includes an elastic amplifier to amplify the base excitation and provide enough kinetic energy to overcome the tristable potential well barriers, thus leading to large amplitude bistable intermotion. They only consider to amplify the vibration displacement of the base but do not consider how to further amplify the vibration amplitude of the cantilever beam. In order to further improve the performance of the energy capture device under weak excitation, a new-type bistable piezoelectric cantilever energy harvester (BPEH) with two dynamic magnifiers (TDMs) is proposed in this paper. It can amplify the amplitude of the low-level base excitation and the vibration amplitude of the fixed end of the piezoelectric cantilever beam at the same time, so as to dramatically improve the output power and effective bandwidth of the piezoelectric energy harvester. Considering the size effect of the tip magnet, the distributed parameter electro-mechanical coupling equation of the bistable piezoelectric energy harvester with two dynamic magnifiers (BPEH + TDM) is established based on the generalized Hamilton principle, and the analytical solution of the energy capture system is derived by using the harmonic balance method. The effects of the distance between the magnets, the mass of the dynamic magnifiers, the load resistance, and the stiffness ratio of the two dynamic magnifiers on the performance of the energy capture system were studied. The results show that compared with the typical bistable piezoelectric energy harvester with a dynamic magnifier, the piezoelectric proposed energy harvester system with a two-spring-mass dynamic magnifier can collect higher output power over a broader frequency band. By reasonably selecting the design parameters of the amplifier, the harvested power can be significantly increased and the effective bandwidth of the harvester can be improved. The mathematical model of the BPEH + TDM is described in Section 2. The harmonic balance method is used for analytical expressions for the steady-state displacement, steady-state output voltage, and power amplitude of the BPEH + TDM in Section 3. The effects of parameter variations of the BPEH + TDM on its dynamic characteristics are numerically investigated in Section 4.

## 2. Mathematical Model of the BPEH + TDM

The BPEH + TDM configuration considered in this paper is schematically shown in Figure 1. The BPEH comprises a piezoelectric cantilever beam and two magnets (denoted as A and B). The piezoelectric cantilever beam is composed of a substrate layer, covered with a pair of piezoelectric layers (PZTs) on both of its surfaces, and poled oppositely in the thickness direction. The two piezoelectric layers are electrically connected in series with a load resistance (*R*), representing the equivalent resistance of a low power electronic device. Magnet A (called the tip magnet) is attached to the tip of the cantilever beam and the external magnet B is fixed at the right wall of the L-shaped frame. The TDM comprises two dynamic magnifiers (denoted as DM1 and DM2), the DM1 is basically a spring (*k*_f_)-mass (*M*_f_) system placed between the fixed end of the piezoelectric beam and the bottom of the L-shaped frame, and the DM2 composed an L-shaped frame and a spring *k*_b,_ and the L-shaped frame is mechanically connected in series with the spring *k*_b_. *M*_f_ and *M*_m_ represent the mass of DM1 and DM2, respectively. The horizontal gap between the tip magnet and magnet B is *d*. Here, *l* and *b* are the length and width of the piezoelectric cantilever beam, respectively; *h*_s_ and *t*_p_ denote the thickness of the substrate layer and the PZTs, respectively; *e* is the eccentricity of the tip magnet.

*v*_*m*_(*t*) and *v*_*b*_(*t*) represent the vibration displacement of the DM2 and the base, respectively. *s* is the coordinate along the neutral axis of the beam, and *v*(*s*, *t*) represents the displacement of the beam at *s* position relative to its fixed end. The constitutive equations of the piezoelectric cantilever beam are assumed as follows:

(1) $$\begin{array}{c} \left.\begin{array}{c} T_{1}^{s}=Y_{s}S_{1}^{s}\\ T_{1}^{p}=Y_{p}\left(S_{1}^{p}-d_{31}E_{3}\right)\\ D_{3}=d_{31}T_{1}+\varepsilon_{33}^{T}E_{3} \end{array}\right\}. \end{array}$$

Here, *Y* is Young's modulus, subscript/superscript *p* and *s* represent the piezoelectric layers and substrate layer, and *S*_1_ and *T*_1_ are the strain and the stress of the beam, respectively. *D*_3_ is the electric displacement and *d*_31_ and *ε*_33_^*T*^ are the piezoelectric constant and dielectric constant, respectively. *E*_3_=−*V*(*t*)/(2*t*_*P*_) is the electric field, in which *V*(*t*) represents the voltage. The strain generated in the piezoelectric beam can be assumed as *S*_1_^*s*^=*S*_1_^*p*^=−*yv*^″^.

The generalized Hamilton's principle of the BPEH + TDM system is as follows:

(2) $$\begin{array}{c} \int_{t_{1}}^{t_{2}}\left[\delta \left(T_{\text{k}}+W_{e}-U_{\text{e}}-U_{\text{m}}-U_{\text{d}}\right)+\delta W\right]\text{d}t=0. \end{array}$$

Here, *T*_k_, *W*_e,_*U*_e_, *U*_m_, *U*_d_, and *W* are the kinetic energy, the electrical energy, the strain energy, the magnetic potential energy, the elastic potential of the dynamic magnifiers, and the external work, respectively. *T*_k_ and *W*_e_ are as follows:

(3) $$\begin{array}{c} T_{k}=\frac{1}{2}\int_{0}^{l}m{\left(\dot{v}+{\dot{v}}_{m}\left(t\right)\right)}^{2}\text{d}s+\frac{1}{2}M_{t}{\left(\dot{v}\left(l,t\right)+e{\dot{v}}^{\prime }\left(l,t\right)+{\dot{v}}_{m}\left(t\right)\right)}^{2}+\frac{1}{2}J{\dot{v}}^{\prime }{\left(l,t\right)}^{2} \end{array}$$

(4) $$\begin{array}{c} W_{e}=\frac{1}{2}Y_{p}bd_{31}\left(h+\frac{t_{p}}{2}\right)V\left(t\right)\int_{0}^{l}v^{\prime \prime }\text{d}s+bl\varepsilon_{33}^{S}\frac{V{\left(t\right)}^{2}}{4t_{p}}. \end{array}$$

Here, *m*=2*ρ*_*p*_*t*_*p*_*b*+*ρ*_*s*_*h*_*s*_*b*, in which *ρ*_*p*_ and *ρ*_*s*_ are the density of the piezoelectric layers and substrate layer, respectively. *M*_t_ is the tip magnet mass and *J* represents the rotary inertia of the tip magnet, *ε*_33_^*s*^ is the permittivity.

*U*_e_ is expressed as follows:

(5) $$\begin{array}{c} U_{\text{e}}=\frac{1}{2}\int_{0}^{l}\left[YI{v^{\prime \prime }}^{2}-Y_{\text{p}}bd_{31}\left(h+\frac{t_{\text{p}}}{2}\right)V\left(t\right)v^{\prime \prime }\right]\text{d}s. \end{array}$$

Here, *h*=(*h*_*s*_/2), *YI*=(2/3)[*Y*_*s*_*bh*^3^+*Y*_*p*_*b*(3*h*^2^*t*_*p*_+3*ht*_*p*_^2^+*t*_*p*_^3^)].

*U*_d_ is expressed as follows:

(6) $$\begin{array}{c} U_{d}=\frac{1}{2}k_{f}v{\left(0,t\right)}^{2}+\frac{1}{2}k_{b}v_{m}^{2}. \end{array}$$

Here, *k*_f_ and *k*_b_ represent the stiffness of DM1 and DM2, respectively. Considering the eccentricity of the tip magnet, *U*_m_ can be given by the following equation:

(7) $$\begin{array}{c} U_{\text{m}}=\mu_{0}M_{\text{A}}V_{\text{A}}M_{\text{B}}V_{\text{B}}\left\{-{\left(v\left(l,t\right)+\frac{ev^{\prime }\left(l,t\right)}{\sqrt{1+v^{\prime }{\left(l,t\right)}^{2}}}\right)}^{2}\right.+2{\left[d+e\left(1-\frac{1}{\sqrt{1+v^{\prime }{\left(l,t\right)}^{2}}}\right)\right]}^{2}\\ \left.-3\left[d+e\left(1-\frac{1}{\sqrt{1+v^{\prime }{\left(l,t\right)}^{2}}}\right)\right]\left(v\left(l,t\right)+\frac{ev^{\prime }\left(\text{l,t}\right)}{\sqrt{1+v^{\prime }{\left(l,t\right)}^{2}}}\right)v^{\prime }\left(l,t\right)\right\}\\ 4\pi \sqrt{1+v^{\prime }{\left(l,t\right)}^{2}}{\left\{{\left[d+e\left(1-\frac{1}{\sqrt{1+v^{\prime }{\left(l,t\right)}^{2}}}\right)\right]}^{2}+{\left(v\left(l,t\right)+\frac{ev^{\prime }\left(l,t\right)}{\sqrt{1+v^{\prime }{\left(l,t\right)}^{2}}}\right)}^{2}\right\}}^{5/2}. \end{array}$$

Here, *μ*_0_=4*π* × 10^−7^*H* · *m*^−1^ is the magnetic permeability constant. *M*_A_ (*M*_B_) and *V*_A_ (*V*_B_) are the magnetization intensity and volume of the magnet A (B), respectively.

Using the Galerkin approach, *v*(*s*, *t*) can be written as follows:

(8) $$\begin{array}{c} v\left(s,t\right)=\phi_{r}\left(s\right)\eta_{r}\left(t\right). \end{array}$$

Here, *φ*_*r*_(*s*) and *η*_*r*_(*t*) represent the R-order mode shape function and the generalized mode coordinates of the beam, respectively.

The modal shape function satisfies the following orthogonal relations:

(9) $$\begin{array}{c} \int_{0}^{l}\phi_{s}\left(s\right)m\phi_{r}\left(s\right)\text{d}s+\phi_{s}\left(l\right)M_{t}\phi_{r}\left(l\right)+\phi_{s}\left(l\right)M_{t}e\phi_{r}^{\prime }\left(l\right)+\phi_{s}\left(0\right)M_{f}\phi_{r}\left(0\right) \end{array}$$

(10) $$\begin{array}{c} \int_{0}^{l}\frac{{\text{d}}^{2}\phi_{s}\left(s\right)}{\text{d}s^{2}}YI\frac{{\text{d}}^{2}\phi_{r}\left(s\right)}{\text{d}s^{2}}\text{d}s+\phi_{s}\left(0\right)k_{f}\phi_{r}\left(0\right)=\omega_{r}^{2}\delta_{rs}. \end{array}$$

Here, *δ*_*rs*_ represents the Kronecker delta. $\omega_{r}=\lambda_{r}^{2}\sqrt{YI/\left(ml^{4}\right)}$ represents the resonance frequency of the *r*-th mode, in which *λ*_*r*_ is the eigenvalue. The calculation process of the *λ*_*r*_ is described in the literature [33, 34].

Substituting equation (8) into (7), the Taylor's expansion of *U*_*m*_ at *η*(*t*)=0 can be expressed as follows:

(11) $$\begin{array}{c} U_{m}=k_{0}-\frac{1}{2}k_{1}\eta_{1}^{2}+\frac{1}{4}k_{2}\eta_{1}^{4}+o\left(\eta_{1}^{5}\right). \end{array}$$

Here, *k*_0_=2*κ*/*d*^3^,

(12) $$\begin{array}{c} k_{1}=\frac{\kappa \left(10q_{1}+2d^{2}\phi_{1}^{\prime }{\left(l\right)}^{2}+2q_{2}\right)}{d^{5}},\\ k_{2}=\frac{\kappa \left[8d^{2}q_{3}+35q_{1}^{2}+10\left(d^{2}\phi_{1}^{\prime }{\left(l\right)}^{2}+q_{2}\right)q_{1}+\left(3d^{2}\phi_{1}^{\prime }{\left(l\right)}^{4}+2q_{2}\phi_{1}^{\prime }{\left(l\right)}^{2}+4q_{4}\right)d^{2}\right]}{d^{7}},\\ q_{1}=de\phi_{1}^{\prime }{\left(l\right)}^{2}+e^{2}\phi_{1}^{\prime }{\left(l\right)}^{2}+2e\phi_{1}\left(l\right)\phi_{1}^{\prime }\left(l\right)+\phi_{1}{\left(l\right)}^{2},\\ q_{2}={\left(e\phi_{1}^{\prime }\left(l\right)+\phi_{1}\left(l\right)\right)}^{2}-2\;\;de\;\;\phi_{1}^{\prime }{\left(l\right)}^{2}+3\;\;d\left(e\phi_{1}^{\prime }\left(l\right)+\phi_{1}\left(l\right)\right)\phi_{1}^{\prime }\left(l\right),\\ q_{3}=2.5\left(0.75\;\;de\;\;\phi_{1}^{\prime }{\left(l\right)}^{4}+0.75e^{2}\phi_{1}^{\prime }{\left(l\right)}^{4}+e\phi_{1}\left(l\right)\phi_{1}^{\prime }{\left(l\right)}^{3}\right),\\ q_{4}=\left(e\phi_{1}^{\prime }\left(l\right)+\phi_{1}\left(l\right)\right)e\phi_{1}^{\prime }{\left(l\right)}^{3}-1.5\;\;de\;\;\phi_{1}^{\prime }{\left(l\right)}^{4}+0.5e^{2}\phi_{1}^{\prime }{\left(l\right)}^{4}\\ -3\left[-0.5\;\;de\;\;\phi_{1}^{\prime }{\left(l\right)}^{3}+0.5e\phi_{1}^{\prime }{\left(l\right)}^{2}\left(e\phi_{1}^{\prime }\left(l\right)+\phi_{1}\left(l\right)\right)\right]\phi_{1}^{\prime }\left(l\right),\\ \kappa =\frac{\mu M_{A}V_{A}M_{B}V_{B}}{4\pi },\\ \delta W=\delta v_{m}{\ddot{v}}_{b}\left(M_{m}+M_{t}+ml+M_{f}\right)+\delta \eta \left(t\right){\ddot{v}}_{b}\left(M_{t}\phi_{1}\left(l\right)+m\int_{0}^{l}\phi_{1}\left(s\right)\text{d}s+M_{t}e\phi_{1}^{\prime }\left(l\right)+M_{f}\phi_{1}\left(0\right)\right). \end{array}$$

The external virtual work can be defined as follows.

Substituting equation (8) into (2) and considering only the 1st order mode, Lagrange's equation for the BPEH + TDM system is given by the following equation:

(13) $$\begin{array}{c} \left\{\begin{array}{c} \frac{\text{d}}{\text{d}t}\left(\frac{\partial L}{\partial {\dot{v}}_{m}}\right)-\frac{\partial L}{\partial v_{m}}+\frac{\partial W}{\partial v_{m}}=0,\\ \frac{\text{d}}{\text{d}t}\left(\frac{\partial L}{\partial \dot{\eta }}\right)-\frac{\partial L}{\partial \eta }+\frac{\partial W}{\partial \eta }=F\left(t\right),\\ \frac{\text{d}}{\text{d}t}\left(\frac{\partial L}{\partial \dot{V}}\right)-\frac{\partial L}{\partial V}+\frac{\partial W}{\partial V}=Q\left(t\right). \end{array}\right. \end{array}$$

Here, $F_{1}\left(t\right)=-2\xi_{1}\omega_{1}{\dot{\eta }}_{1}\left(t\right)$ is the generalized dissipative force, *ξ*_1_ is the damping ratio, and *Q*(*t*)=*V*(*t*)/*R* represents the generalized output charge.

The electro-mechanical coupling equations of the BPEH + TDM system can be obtained by using the following equation:

(14) $$\begin{array}{c} \left\{\begin{array}{c} M_{0}{\ddot{\eta }}_{1}\left(t\right)+M_{1}{\ddot{v}}_{m}\left(t\right)+k_{b}v_{m}=-M_{1}{\ddot{v}}_{b}\left(t\right),\\ {\ddot{\eta }}_{1}\left(t\right)+2\xi_{1}\omega_{1}{\dot{\eta }}_{1}\left(t\right)+\omega_{1}^{2}\eta_{1}\left(t\right)-k_{1}\eta_{1}\left(t\right)+k_{2}\eta_{1}{\left(t\right)}^{3}-\theta_{1}V\left(t\right)+M_{0}{\ddot{v}}_{m}\left(t\right)=-M_{0}{\ddot{v}}_{b}\left(t\right),\\ C_{p}\dot{V}\left(t\right)+\frac{V\left(t\right)}{R}+\theta_{1}{\dot{\eta }}_{1}\left(t\right)=0. \end{array}\right. \end{array}$$

Here, *M*_0_=*m*∫_0_^*l*^*φ*_1_(*s*)d*s*+*M*_*t*_*φ*_1_(*l*)+*M*_*t*_*eφ*_1_′(*l*)+*M*_*f*_*φ*_1_(0), *M*_1_=*ml*+*M*_*t*_+*M*_*f*_+*M*_*m*_, *ω*_1_^2^=*YI*∫_0_^*l*^*φ*_1_^″^(*s*)^2^d*s*+*k*_*f*_*φ*_1_(0)^2^, *θ*_1_=*Y*_*p*_*bd*_31_(*h*+(*t*_*p*_/2))∫_0_^*l*^*φ*_1_^″^(*s*)d*s*, *C*_*p*_=*blε*_33_^*S*^/2*t*_*p*_. Here, *ω*_1_^2^=*YI*∫_0_^*l*^*φ*_1_^'′^d*s*, *g*_0_=*mg*∫_0_^*l*^*φ*_1_(*s*)d*s*+*M*_*t*_*gφ*_1_(*l*), Γ_1_=*m*∫_0_^*l*^*φ*_1_(*s*)*ds*+*M*_*t*_(*φ*_1_(*l*)+*eφ*_1_′(*l*)), *θ*_1_=*Y*_*p*_*bd*_31_(*h*+(*t*_*p*_/2))∫_0_^*l*^*φ*_1_(*s*)d*s*, and *C*_*p*_=*blε*_33_^*s*^/2*t*_*p*_.

The excitation acceleration is assumed to be ${\ddot{v}}_{b}\left(t\right)={\ddot{v}}_{b}cos\left(\omega_{e}t\right)$, where ${\ddot{v}}_{b}$ denotes the excitation amplitude, *ω*_*e*_ denotes the circular frequency, and *C*_p_ denotes the capacitance. Introducing the dimensionless parameters *x*=*η*_1_/*l*, *V*_*m*_=*v*_*m*_/*l*, *V*_*b*_=*v*_*b*_/*l*, $\ddot{V}=\left(VC_{p}/l\theta_{1}\right)$, *τ*=*ω*_1_*t*, equation (14) can be rewritten as the following equation in the dimensionless form:

(15) $$\begin{array}{c} \left\{\begin{array}{c} \frac{M_{1}-M_{0}^{2}}{K_{b}}x^{\left(4\right)}+\frac{2M_{1}\xi_{1}}{K_{b}}x^{\left(3\right)}+\frac{M_{1}\left(1-K_{1}\right)+K_{b}}{K_{b}}\ddot{x}+2\xi_{1}\dot{x}+\left(1-K_{1}\right)x+K_{2}x^{3}\\ +\frac{M_{1}K_{2}}{K_{b}}\left(6x{\dot{x}}^{2}+3x^{2}\ddot{x}\right)-\frac{M_{1}\Theta }{K_{b}}\ddot{V}-\Theta \ddot{V}=F\;\;\cos\left(\omega \tau \right),\\ \ddot{V}+\alpha \ddot{V}+\dot{x}=0. \end{array}\right. \end{array}$$

Here, *K*_*b*_=*k*_*b*_/*ω*_1_^2^, *K*_1_=*k*_1_/*ω*_1_^2^, *K*_2_=*k*_2_*l*^2^/*ω*_1_^2^, Θ=*θ*_1_^2^/*C*_*p*_*ω*_1_^2^, *α*=1/*C*_*p*_*R*_*L*_*ω*_1_, $F=-M_{0}\overset{-}{v_{b}}/\omega_{1}^{2}l$.

## 3. Harmonic Balance Analysis

The solution of equation (15) is assumed to be

(16) $$\begin{array}{c} \left\{\begin{array}{c} x=A\left(\tau \right)+B\left(\tau \right)\sin\left(\omega \tau \right)+C\left(\tau \right)\cos\left(\omega \tau \right),\\ \bar{V}=D\left(\tau \right)\sin\left(\omega \tau \right)+E\left(\tau \right)\cos\left(\omega \tau \right). \end{array}\right. \end{array}$$

Here, *A*, *B*, *C*, *D,* and *E* are undetermined coefficients, so the displacement amplitude can be expressed as $a=\sqrt{B^{2}+C^{2}}$ and the output voltage amplitude can be expressed as $u=\sqrt{D^{2}+E^{2}}$.

Substituting equation (16) into (15), let the constant terms on both sides of the equation and the coefficients of sin(*ωτ*) and cos(*ωτ*) consistent and ignoring the high-order harmonic term and partial zero term, we can obtain the following equations:

(17) $$\begin{array}{c} Z_{1}\ddot{A}+2\xi_{1}\dot{A}+\left(1-K_{1}\right)A+K_{2}A^{3}+\frac{3}{2}K_{2}A\left(B^{2}+C^{2}\right)=0, \end{array}$$

(18) $$\begin{array}{c} Z_{1}\left(\ddot{B}-2\omega \dot{C}\right)+2\xi_{1}\dot{B}+Z_{2}C+Z_{3}B+Z_{4}D=0, \end{array}$$

(19) $$\begin{array}{c} Z_{1}\left(\ddot{C}-2\omega \dot{B}\right)+2\xi_{1}\dot{C}+Z_{3}C-Z_{2}B+Z_{4}E-F=0, \end{array}$$

(20) $$\begin{array}{c} \dot{D}-\omega E+\alpha \;\;D+\dot{B}-\omega C=0, \end{array}$$

(21) $$\begin{array}{c} \dot{E}+\omega \;\;D+\alpha E+\dot{C}+\omega B=0. \end{array}$$

Here,

(22) $$\begin{array}{c} Z_{1}=\frac{K_{1}M_{1}+K_{b}}{K_{b}},\\ Z_{2}=\frac{2\xi_{1}M_{1}}{K_{b}}\omega^{3}-2\xi_{1}\omega ,\\ Z_{3}=\frac{M_{1}-M_{0}^{2}}{K_{b}}\omega^{4}-\frac{\left(1-K_{1}\right)M_{1}+K_{b}}{K_{b}}\omega^{2}+1-K_{1}+K_{2}\left(3A^{2}+\frac{3}{4}a^{2}\right)-\frac{K_{2}M_{1}}{K_{b}}\omega^{2}\left(3A^{2}+\frac{3}{4}a^{2}\right),\\ Z_{4}=\frac{\Theta M_{1}}{K_{b}}\omega^{2}-\Theta . \end{array}$$

As the undetermined coefficients *A*, *B*, *C*, *D,* and *E* in equations (17)–(21) change slowly, it can be considered that

(23) $$\begin{array}{c} \left\{\begin{array}{c} \frac{dA}{d\tau }=\frac{dB}{d\tau }=\frac{dC}{d\tau }=\frac{d\;\;D}{d\tau }=\frac{dE}{d\tau }=0,\\ \frac{d^{2}A}{d\tau^{2}}=\frac{d^{2}B}{d\tau^{2}}=\frac{d^{2}C}{d\tau^{2}}=\frac{d^{2}D}{d\tau^{2}}=\frac{d^{2}E}{d\tau^{2}}=0,\\ \frac{d^{3}A}{d\tau^{3}}=\frac{d^{3}B}{d\tau^{3}}=\frac{d^{3}C}{d\tau^{3}}=0,\\ \frac{d^{4}A}{d\tau^{4}}=\frac{d^{4}B}{d\tau^{4}}=\frac{d^{4}C}{d\tau^{4}}=0. \end{array}\right. \end{array}$$

Using equations (20) and (21), we obtain the following equations:

(24) $$\begin{array}{c} D=\frac{\omega }{\omega^{2}+\alpha^{2}}\left(\alpha C-\omega B\right), \end{array}$$

(25) $$\begin{array}{c} E=-\frac{\omega }{\omega^{2}+\alpha^{2}}\left(\omega C+\alpha B\right). \end{array}$$

Then, substituting formulas equations (20) and (21) into equations (18) and (19), respectively, we obtain the following equations:

(26) $$\begin{array}{c} B=-\frac{F\left(Z_{2}+Z_{4}\left(\alpha \omega /\omega^{2}+\alpha^{2}\right)\right)}{{\left(Z_{3}-\left(Z_{4}\omega^{2}/\left(\omega^{2}+\alpha^{2}\right)\right)\right)}^{2}+{\left(Z_{2}+\left(Z_{4}\alpha \omega /\left(\omega^{2}+\alpha^{2}\right)\right)\right)}^{2}}, \end{array}$$

(27) $$\begin{array}{c} C=-\frac{F\left(\left(Z_{4}\omega^{2}/\left(\omega^{2}+\alpha^{2}\right)\right)-Z_{3}\right)}{{\left(Z_{3}-\left(Z_{4}\omega^{2}/\left(\omega^{2}+\alpha^{2}\right)\right)\right)}^{2}+{\left(Z_{2}+\left(Z_{4}\alpha \omega /\left(\omega^{2}+\alpha^{2}\right)\right)\right)}^{2}}. \end{array}$$

Therefore, the displacement amplitude and the voltage amplitude can be expressed as follows:

(28) $$\begin{array}{c} a^{2}\left[{\left(Z_{2}+Z_{4}\frac{\alpha \omega }{\omega^{2}+\alpha^{2}}\right)}^{2}+{\left(Z_{3}-Z_{4}\frac{\omega^{2}}{\omega^{2}+\alpha^{2}}\right)}^{2}\right]=F^{2}. \end{array}$$

Here, the steady-state displacement response amplitude *a* can be obtained by equation (23), and the steady-state output voltage amplitude and output power amplitude can then be expressed in the following forms:

(29) $$\begin{array}{c} u=\left(\frac{\omega }{\sqrt{\omega_{2}+\alpha^{2}}}\right)a, \end{array}$$

(30) $$\begin{array}{c} P=\frac{l^{2}\theta_{1}^{2}u^{2}}{C_{p}^{2}R}. \end{array}$$

## 4. Results and Discussion

In this section, we numerically investigate the effects of the magnet spacing, the mass of the base dynamic magnifier *M*_m_, the load resistance, the stiffness ratio of the *k*_f_ to *k*_b_, and the mass ratio of the *M*_f_ to *M*_t_ on the dynamic characteristics of the BPEH + TDM system. The geometric and material properties are as follows [35]: *l*=75*mm*, *b*=20*mm*, *h*_*s*_=0.2*mm*, *Y*_*s*_=70*Gpa*, *ρ*_*s*_=2700kg/m^3^, *M*_*t*_=10 × 10^−3^*kg*, *M*_*m*_=0.18*kg*, *M*_*f*_=16.5 × 10^−3^*kg*, *k*_*f*_=10.2*KN* · *m*, *k*_*b*_=15.8*KN* · *mM*_*A*_=*M*_*B*_=1.22 × 10^6^*A*/*m*, *V*_*A*_=*V*_*B*_=1 × 10^−6^*m*^3^, *ξ*_1_=0.01. *Y*_*p*_=60.98*Gpa*, *ρ*_*s*_=7750*kg*/*m*^3^, *d*_31_=−1.71 × 10^−10^*C*/*N*, *ε*_33_^*s*^=1.33 × 10^−8^*F*/*m*.

In Figures 2 and 3, we define three bistable piezoelectric energy harvester (BPEH) calculation models, namely, BPEH + DM1 (BPEH with a dynamic amplifier placed between the fixed end of the piezoelectric beam and the base structure), BPEH + DM2 (BPEH with a dynamic amplifier placed between the BPEH and the base structure), and BPEH + TDM (BPEH with DM1 and DM2 amplifiers).  Figure 2 depicts variations of displacement and output power versus excited frequency for different calculation models when *d* = 16 mm, *M*_t_ = 10 g, *M*_f_ = 16.5 g, and *R* = 300 k*Ω*. It shows that among the three calculation models, the peak displacement and peak power of the interwell motion of BPEH + TDM are the highest, and its frequency bandwidth is also the widest. When magnet spacing *d* increases to 20 mm, it can be seen from Figure 3 that the peak displacement and peak output power of the three calculation models increase significantly, however, the interwell frequency bandwidth decreases.

Figures 4–6 show the steady-state amplitude response curves of the BPEH + TDM interwell motion displacement and output power with the variation of the base amplifier mass *M*_m_ for different stiffness ratios of *k*_f_ to *k*_b_ when excited frequency *ω*=1.4, *ω*=1.7, and *ω*=2. As can be seen from Figure 4, when excited frequency *ω*=1.4, the displacement amplitude and output power amplitude of the BPEH + TDM first increase to extreme values as the mass of the base amplifier *M*_m_ gradually increases, then rapidly decreases, and finally, tend to be stable in a small range, and there exists an optimal mass of the base amplifier mass *M*_m_ value which maximizes the displacement amplitude and output power amplitude of the system, and the optimal *M*_m_ value increases with the stiffness ratio of *k*_f_ to *k*_b_ increasing.

Figures 5 and 6 show that when the excitation frequency increases, with the gradual increase of the *M*_m_, the displacement amplitude and output power amplitude of the BPEH + TDM will first increase to the extreme value, then decreases sharply followed by a slight increase, and finally tend to be stable due to falling into the intrawell. It can also be seen from Figure 4 that with the increase of stiffness ratio *k*_f_/*k*_b_, the optimal value of *M*_m_ increases, and when *M*_m_ reaches the optimal value, the corresponding displacement amplitude and output power amplitude of the BPEH + TDM also increase with the stiffness ratio *k*_f_/*k*_b_ increasing.

Figures 7–9 give the power amplitude variation curve with excited frequency for different values of the mass ratio *M*_f_/*M*_t_ when *M*_m_ = 0.12 kg, *M*_m_ = 0.15 kg and *M*_m_ = 0.18 kg. Figures 7–9 show that when the base amplifier *M*_m_ and magnet spacing *d* are kept constant, the peak output power of the BPEH + TDM increases significantly as the mass ratio of the *M*_f_ to *M*_t_ increases and the excitation frequency at which the system generates peak power decreases. It can also be found from the results of Figures 7–9 that when magnet spacing *d* and mass ratio *M*_f_/*M*_t_ remain unchanged, the peak output power of the BPEH + TDM decreases with the increase of *M*_m_. However, the reduction rate of the peak power slows down as *M*_m_ becomes larger. When *d* = 20 mm, *M*_f_/*M*_t_ = 1.8, taking *M*_m_ = 0.15 kg as examples, the peak power of the BPEH + TDM is 0.069 W, which is 21.6% lower than that of *M*_m_ = 0.12 kg. However, when *M*_m_ increases to 0.18 kg, the corresponding peak power of the BPEH + TDM is decreased by 14.3%, compared with that of *M*_m_ = 0.15 kg.

Figure 10 shows the variation of output power amplitude with load resistance for magnet spacing *d* = 18 mm and *d* = 20 mm. The results show the power amplitude tends to increase at the beginning and decrease afterwards with the increase of load resistance at each excited frequency. Each excitation frequency corresponds to an optimal load resistance to maximize the amplitude of power of the BPEH + TDM, and the optimal load resistance decreases with the increase of excitation frequency. The optimal resistance decreases with the increase of magnet spacing, but the corresponding peak power is significantly higher when the magnet spacing increases.

## 5. Conclusions

In this paper, based on the generalized Hamilton variational principle, considering the size effect and the rotary inertia of the tip magnet, an electro-mechanical coupling equation of the BPEH + TDM system is obtained, and the analytical solution of the equation is obtained by using the harmonic balance method. The effects of magnet spacing, the mass of the base dynamic magnifier *M*_m_, the load resistance, the stiffness ratio of the *k*_f_ to *k*_b_, and the mass ratio of the *M*_f_ to *M*_t_ on the BPEH + TDM system are investigated and the following conclusions were obtained:

1. Increasing the magnet spacing can improve the interwell output power amplitude of the BPEH + TDM system, but the interwell frequency bandwidth decreases.
2. There exists an optimal mass of the base dynamic magnifier to maximize the output power of the BPEH + TDM system, and the optimal value of the base dynamic magnifier mass increases with the increase of stiffness ratio *k*_f_/*k*_b._
3. The peak output power of the BPEH + TDM system increases significantly as the mass ratio of the *M*_f_ to *M*_t_ increases, and the excitation frequency at which the system generates peak power decreases with increasing *M*_f_/*M*_t_. The peak output power of the BPEH + TDM decreases with the increase of *M*_m_. However, the reduction rate of the peak power slows down when *M*_m_ is large.
4. Compared with the BPEH + DM1 system which a dynamic amplifier is placed between the fixed end of the piezoelectric beam and the BPEH + DM2 system which a dynamic amplifier is placed between the BPEH and the base structure, the BPEH + TDM system can produce higher peak output power and wider interwell bandwidth.

In many cases, the excitation of piezoelectric energy capture devices is mostly random. In the future, to further explore the strategy of inducing the multistable energy harvester to vibrate on the high energy orbit for low-level random excitation is of great significance to improve the application of piezoelectric energy harvesting.

## Figures and Tables

**Figure 1:** Schematic of the considered BPEH + TDM.

**Figure 2:** Displacement amplitude (left column) and output power amplitude (right column) versus excitation frequency for: (a) BPEH + DM1. (b) BPEH + DM2. (c) BPEH + TDM when *d* = 16 mm.

**Figure 3:** Displacement amplitude (left column) and output power amplitude (right column) versus excitation frequency for: (a) BPEH + DM1. (b) BPEH + DM2. (c) BPEH + TDM when *d* = 20 mm.

**Figure 4:** (a) Displacement amplitude and (b) output power amplitude versus the mass of the base amplifier *M*_m_ for excited frequency *ω*=1.4 with different value of the stiffness ratio *k*_f_/*k*_b_.

**Figure 5:** (a) Displacement amplitude and (b) output power amplitude versus the mass of the base amplifier *M*_m_ for excited frequency *ω*=1.7 with different value of the stiffness ratio *k*_f_/*k*_b_.

**Figure 6:** (a) Displacement amplitude and (b) output power amplitude versus the mass of the base amplifier *M*_m_ for excited frequency *ω*=2 with different value of the stiffness ratio *k*_f_/*k*_b_.

**Figure 7:** Power frequency response curve in different values of the mass ratio *M*_f_/*M*_t_ for *M*_m_ = 0.12 kg when (a) *d* = 16 mm, (b) *d* = 20 mm.

**Figure 8:** Power frequency response curve in different values of the mass ratio *M*_f_/*M*_t_ for *M*_m_ = 0.15 kg when (a) *d* = 16 mm, (b) *d* = 20 mm.

**Figure 9:** Power frequency response curve in different values of the mass ratio *M*_f_/*M*_t_ for *M*_m_ = 0.18 kg when (a) *d* = 16 mm, (b) *d* = 20 mm.

**Figure 10:** Output power amplitude response of the system with different load resistance: (a) *d* = 18 mm and (b) *d* = 20 mm.

## Data Availability

The data used to support the findings of this study are available from the corresponding author upon request.
